The article "Diagnosis of Chronic Ischemic Heart Disease Using Machine Learning Techniques" was published in 2022. Journal: Comput Intell Neurosci.

# Diagnosis of Chronic Ischemic Heart Disease Using Machine Learning Techniques

**DOI:** 10.1155/2022/3823350

**Published:** 2022-06-14

**Authors:** Shumaila Shehzadi, Muhammad Abul Hassan, Muhammad Rizwan, Natalia Kryvinska, Karovič Vincent

**Affiliations:** ^1^Department of Computer Science, Kinnaird College for Women, Lahore 54000, Pakistan; ^2^Department of Computing and Technology, Abasyn University, Peshawar 25000, Pakistan; ^3^Secure Cyber Systems Research Group, WMG University of Warwick, Coventry CV4 7AL, UK; ^4^Information Systems Department, Faculty of Management Comenius University in Bratislava, Odbojárov 10, 82005 Bratislava 25, Slovakia

## Abstract

Ischemic heart disease (IHD) causes discomfort or irritation in the chest. According to the World Health Organization, coronary heart disease is the major cause of mortality in Pakistan. Accurate model with the highest precision is necessary to avoid fatalities. Previously several models are tried with different attributes to enhance the detection accuracy but failed to do so. In this research study, an artificial approach to categorize the current stage of heart disease is carried out. Our model predicts a precise diagnosis of chronic diseases. The system is trained using a training dataset and then tested using a test dataset. Machine learning methods such as LR, NB, and RF are applied to forecast the development of a disease. Experimental outcomes of this research study have proven that our strategy has excelled other procedures with maximum accuracy of 99 percent for RF, 97 percent for NB, and 98 percent for LR. With such high accuracy, the number of deaths per year of ischemic heart disease will be slightly decreased.

## 1. Introduction

Atherosclerosis is a prominent cause of death globally. Professionals, on the other hand, typically have trouble detecting heart illness owing to a high degree of ambiguity and a risk factor [1]. When a heart attack happens, speed is of the essence in saving the patient's life and avoiding heart failure. According to the World Health Organization, 12 million people die each year from cardiovascular disease. Clinical call support systems may assist patients to make better judgments than medical examiners [2, 3]. In a world of cloud computing and fog computing, it is nearly impossible to extract healthcare demands without complete, comprehensive, and associated health data, and the security of this data is still another challenge [4–7]. Patient feedback is helpful in the pattern classification process, which establishes a patient's health status and degree of sickness. An expert system might use this information to determine whether or not a patient is suffering from illness. The doctor makes medical decisions based on accurate signs or measurements [8, 9]. There has been great growth in today's contemporary period, for example, in the use of information technology and the Internet of Things (IoT) in diagnostic medicine, sickness prevention, and patient satisfaction [10–14].

W.H.O. and World Bank investigations reveal that more than a few individuals suffer from ischemic heart attacks [15]. Most prosperous countries have a lower incidence of ischemic heart disease than undeveloped ones. As a consequence of the complexity and unpredictability of these sectors, smart structures, such as the fuzzy system and artificial neural network, as well as genetic algorithms, have been created. Smoking, cholesterol, blood pressure, diabetes, sex, and age are the key risk factors for ischemic heart disease [16]. Heart disease is difficult to identify because of the numerous unknown risk factors [17]. When diagnosing a patient's cardiac condition, a doctor must take into consideration a huge number of criteria. This implies that professionals need a technology that can take these risk factors into account and foresee the results [18]. The fact that these computer areas are complicated and sporadic, as well as the utilization of specialist systems, such as mathematical logic, neural networks, and evolutionary algorithms, has been well known to us for some time. Fuzzy logic is a strong technique of thinking that can handle difficult outcomes satisfactorily [19]. Novel fuzzy expert systems enable patients to make choices more helpful than medical examiners. It is a health information management system designed to give medical decision assistance to physicians and healthcare practitioners. The working principle of fuzzy logic system is that the patient should know about his medical health history (data) in order to make proper choices to improve patient health [18]. Novel fuzzy expert systems construct the rules depending upon input qualities and offer results according to them [20]. The IF-Then statements make up the majority of the rule-based knowledge network. The majority of the time, the data are linked to these laws. If the pain intensity is high, for example, the alert system will ring. The knowledge area contains information on the method's principles, while the illusion engine mixes the rules with patient data, and the feedback mechanism informs users of the method's outcomes. It is feasible that data-driven fuzzy logic might assist clear up the ambiguity in demand infrastructure [21]. A number of key approaches and processes have enabled patient diagnosis of disease and pain [14, 22–25]. The formal rules classification is pretty precise when it comes to prognostic price and diagnostic accuracy [26, 27]. Based on the necessity for this critical tool, we designed an expert technique to diagnose heart disease. The fuzzy logic framework was created. Using this fuzzy medical expert system, early findings reveal that it performs substantially better than an expert, with an accuracy rate of roughly 94 percent.  Table 1 provides the definition of abbreviations used in this research investigation. The main motivation behind this research study is as follows:

- To develop an accurate model with higher accuracy, as can be seen in Table 2, previously implemented models did not achieve maximum accuracy mark
- To deploy intelligent classification methods and separate data accordingly

Remaining of the paper is arranged as follows. As a consequence, and an examination of the literature, ischemic heart disease may be identified, and these traits are discussed in Section 2.  Section 3 offers an approach for developing artificial systems. In Section 4, system testing and results are reported, as well as a comparison to earlier investigations. In Section 5, the paper's findings and future directions are explored.

## 2. Literature Review

Researchers have utilized a wide range of data processing technologies in the past to diagnose cardiac disease in various ways. New data processing approaches are being utilized to diagnose cardiac problems, and these methods can be implemented to identify the disease on time.

Automatic heart disease detection employing an artificial immune recognition system (AIRS) with a fuzzy resource allocation mechanism and k-nan (nearest neighbor) based weighted preprocessing classification algorithms are employed for most clinical diagnoses in coronary disease [31, 34]. When analysing the publishing aspects associated with the graduation application, a variety of methodologies were used, including the utilization of data from the UCI machine learning library to achieve high grading accuracies. With ToolDiag, RA obtained 50.00 percent accuracy using the IB1-4 algorithm. Utilizing InductH, WEKA, RA has a rating accuracy of 58.5 percent, whereas using the RBF, ToolDiag, RA has a rating accuracy of 60.00 percent [28]. ToolDiag employed the MLP + BP algorithm, which had a success rate of up to 65%. WEKA and K∗, T2, 1R, IB1c, and RA had classification accuracies of 68.10 percent, 71.40 percent, 74.00 percent, and 76.70 percent, respectively. Robert Detrano utilized a logistic regression approach and got a 77.0 percent classification accuracy. A heart disease fuzzy expert system diagnosis is proposed in the year 2007, where the fuzzy system of experts is utilized to evaluate patients' coronary heart disease risk (CHD) [10]. The machine predicted the danger ratio and may propose one of three outcomes: (1) residing inside a regular method, (2) nourishment, and (3) pharmaceutical treatment. In addition, 79 percent of the outcomes are matched with the expert. For any medical therapy or medical problem, survival prediction after a heart attack from a hospital using a data mining approach and representing a decision tree with data from a service or photocopy of reports may be swiftly accomplished [30, 33]. Cardiologists may use data mining methods to estimate patient survival and adjust operations appropriately. A comparison of normal research and data mining studies revealed the use of the data mining technique to quantity filtering and validated the relevance or influence of data and variables under certain settings. A comparison of conventional research and data mining analysis revealed the impact of the variable-sorting data mining procedure, and we were able to quickly determine the importance or effect of the data and variables on the study's criteria.

Coactive neuro-fuzzy inference system (CANFIS) was utilized to predict heart diseases [29, 36]. By combining and integrating the genetic algorithm of the neural network, adaptive capabilities, and the recirculation qualitative method, the CANFIS model was able to identify illness occurrence. The CANFIS model's performance was evaluated based on training results and classification accuracy. The CANFIS model shows potential in terms of forecasting cardiac disease based on performance.

Using feature extraction and data mining feature selection technologies, an effective framework for heart disease classification is provided [37]. In the categorization of cardiovascular data, a high-dimensional data collection is employed during the preprocessing step of data mining. This ruthless data gathering is made up of repetitious and incomprehensible information. To achieve classification accuracy, we must remove redundant and unnecessary data. Dimensional reduction is a method for reducing high-dimensional data to lower-dimensional data with specified constraints. Heart attacks may be readily anticipated thanks to a mechanism integrated into the system. This technique is used to quickly predict heart disease [32, 38]. The architecture is designed using primary variable analyses (PCA) to separate the features. With the suitable constraint, the statistical model is computed to choose the right characteristics. The suggested work attempts to increase the efficiency, accuracy, and speed of the process. This may be expanded in applications including information storage, picture recognition, and pattern matching [9, 39].

Fuzzy classification and data mining techniques are used to accurately diagnose heart disease [40]. Unstructured data have been discovered as enormous datasets in medical history, and it is predicted that data produced with diverse features may be analysed to forecast and offer information for a cardiac patient's diagnosis. To anticipate people with heart disease, big data have been employed in a variety of circumstances. Data complexity, on the other hand, has not been removed by the data mining tools used by many writers. To reduce ambiguity, a membership feature with a computed value was designed and deployed, and fuzzified data were utilized to forecast individuals with heart disease. In addition, patients should be identified based on characteristics collected from the medical profession. The fuzzy K-NN classifier was built to differentiate training and test data belonging to different classes based on their minimum distance to the Euclidean. In comparison to other classifiers that use parametric approaches, the fuzzy K-NN classifier fits well.

Using a *k*-nearest neighbor algorithm and a simple patient health metric, the heart patient prediction method also offers a screening approach for cardiovascular illness based on real clinical evidence [41]. The *K*-nearest neighbors approach was utilized. A total of 450 papers were prepared and utilized, each of which included the study's criteria. There are 36 types of diseases in the HKH data collection, 29 of which are cardiovascular-related illnesses and 7 of which are not.

## 3. Material and Methods

The suggested research investigates performance analysis to predict cardiac disease. The goal of this research is to accurately predict whether or not the patient has heart disease. The input values from the patient's health report are entered by the health professional. The information is incorporated into a model that forecasts the likelihood of developing heart disease.

### 3.1. Enterprise of the Study

The dataset for this study was gathered via an online dataset platform (Kaggle), and then, conventional statistical measurements (Mean, Median, and Mode) were used to address missing data. Machine learning algorithms, such as logistic regression, naive Bayes, and random forest, are used to classify data towards the conclusion.

### 3.2. Data Collection

All published investigations are based on a subset of the database's 14 features [42]. We utilized the previously processed UCI Cleveland dataset, which is also accessible on Kaggle.  Table 3 provides a detailed description of the 14 criteria used in the planned research.

### 3.3. Preprocessing of Data

After the cleansing of the dataset, the analysis of data attribute and their purpose phase is begun. The total number of occurrences of risk rate attribute with 1 value is 165 and 207 with gender attribute while 138 and 96 (gender attribute) with a value of 0. Pandas is a Python-based data exploration program that is a delight to use. Graphs may be made using Matplotlib, and NumPy is a Python module that enables you to conduct scientific operations swiftly and efficiently with NumPy.

### 3.4. Frequency of Data Set Attributes

A data set's frequency is displayed in this section. Barrels representing the categories of old peak data, age, and red blood pressure are depicted in Figures 1–3. On the *y*-axis, it represents the number of entities. A fraction of each segment's total results is provided as well. According to Figure 1, each patient has a greater blood pressure rate than the other patients, which is symptomatic of cardiac sickness.

### 3.5. Data Encoding Categorical Features

The data were used to produce train and test data. In the same way that learning criteria are applied to training data, they are also used to test data. The encoding technique is used to encrypt categorical information. An estimator builds a transformer to convert object and float data types to integers as part of his training. The estimator performs both data preparation and machine learning model training transformations in a transformation specification. Python's fit tool is used to convert the ML algorithm into a vector matrix, which needs the *X* train and projected data set as inputs.

### 3.6. Training and Testing Dataset

During this phase, many models are trained using various classification approaches, such as the NB, RF, and LR classifiers. Both the input and output variables for a machine learning method must be integer quantities on the same scale. Category and string data must also be translated to numerical data of the same scale as part of the data conversion process. To avoid data loss during the decoding process, data are separated into train and test sets before decoding. Training data are often separated into cross-validation data and reanalysed. 70% of the data are utilized in training, whereas 30% are used in research.

### 3.7. Classification

The features indicated in Table 3 are used as input by ML algorithms such as random forest, logistic regression, and naive Bayes classification techniques [43]. Approximately 70% of the input data are utilized for training, with the remaining 30% for testing. This is the dataset that is used to train a model, also known as the training dataset. When a new model is being trained, it should perform well on a test dataset. As previously stated, the accuracy, precision, recall, and F-measure scores are used to calculate and analyse the performance of each approach. The following is a list of the various algorithms investigated in this study.

### 3.8. Logistic Regression

Logistic regression is the method of choice for binary classification problems. The logistic function is used in logistic regression to compress the result of a linear equation between 0 and 1. Because it includes 13 independent variables, logistic regression is effective for categorization. Logit regression is a machine learning-based categorization technique (ML). It uses logistic functions to represent the results of a single experiment [44].

(1) $$\begin{array}{c} f\left(x\right)=\frac{1}{1+e^{-x}},\\ h\theta \left(x\right)=\frac{L}{1+e^{-k\left(x-x_{0}\right)}}. \end{array}$$

### 3.9. Naive Bayes

The naive Bayes algorithm is based on the Bayes algorithm. The independence of a dataset is the most important assumption to make while categorizing it. It is simple to predict and holds well assuming independence. The Bayesian technique is based on Bayes' theorem and assumes that each pair of attributes is independent. Spam filtering and document classification, for example, are two real-world cases where naive Bayes classifiers are useful. Equation (2) explains how to get the posterior probability of an event (*A*) given a prior probability of an event B using the Bayes theorem.

(2) $$\begin{array}{c} P\left(y\right)=P\left(C_{i}|x_{1},x_{2},..,x_{n}\right)=\frac{P\left(x_{1},x_{2},..,x_{n}|C_{i}\right).P\left(C_{i}\right)}{P\left(x_{1},x_{2},..,x_{n}\right)}\;\text{for }1\leq i\leq k. \end{array}$$

### 3.10. Random Forest

Random forest algorithms are used for both classification and regression. It creates a tree out of the data and forecasts the future in order to make predictions. Despite the fact that the random forest approach may be used to large datasets, the same results can be reached even when large amounts of data include blank values. The constructed decision tree samples may be saved and used on more data. Create the random forest first, and then use the classifier you created in the first step to produce a prediction.

### 3.11. Confusion Matrix of Training Dataset

As a heat map, the confusion matrix makes more sense as a heat map than as an array. A Sci-kit-learn library function is used to plot an uncertainty matrix. An uncertainty matrix is shown to categorize data points that have been mistakenly labelled. The model can correctly predict or differentiate between the groups, as seen in the uncertainty matrix. TP, FP, TN, and FN are combined in this situation. Figures 4 and 5 exhibit the confusion metric for three machine learning algorithms: NB, LR, and RF.

### 3.12. Normalization of Dataset

The process of transforming floating point data to values between 0 and 1 is known as normalization. In order to train algorithms effectively, input feature data are often standardized. The normalized metrics of potential machine learning algorithms such as NB, LR, and RF are given in Figures 5 and 6.

## 4. Result and Analysis

This section discusses the results of random forest, naive Bayes, and logistic regression. The accuracy score, precision (P), recall (R), and F-measure are used to evaluate the algorithm's performance. Precision is used to determine whether or not a positive analysis is accurate. Recall is a metric for how many correct genuine positives there were (or recall score). The F score is a precision metric.

This section presents the output of ML algorithms such as RF, LR, and NB for identifying negative cases. In each situation, the percentage of both truth and classifiers is correct.

TP (true positive): the patient has the disease, and the test is positive derived from equation (3)

TN (true negative): the patient does not have the disease, and the test is negative derived from equation (4)

FP (false positive): the patient does not have the disease, but the test is positive derived from equation (5)

FN (false negative): the patient has the disease but the test is negative derived from equation (6)

(3) $$\begin{array}{c} \text{TP}=\frac{\text{TP}}{\text{TP}+\text{FN}}, \end{array}$$

(4) $$\begin{array}{c} \text{TN}=\frac{\text{TN}}{\text{TP}+\text{FN}}, \end{array}$$

(5) $$\begin{array}{c} \text{FP}=\frac{\text{FP}}{\text{TP}+\text{FP}}, \end{array}$$

(6) $$\begin{array}{c} \text{FN}=\frac{\text{FN}}{\text{TP}+\text{FN}}, \end{array}$$

(7) $$\begin{array}{c} \text{Accuracy}=\frac{\text{TP}+\text{TN}}{\text{TP}+\text{FN}+\text{FP}+\text{TN}}, \end{array}$$

(8) $$\begin{array}{c} F1\text{ score}=\frac{2{\;}^{*}\text{Precision}{\;}^{*}\text{Recall}}{\text{Precision}+\text{Recall}}, \end{array}$$

(9) $$\begin{array}{c} \text{Recall}=\frac{\text{TP}}{\text{TP}+\text{FN}}, \end{array}$$

(10) $$\begin{array}{c} \text{Precision}=\frac{\text{TP}}{\text{TP}+\text{FP}}. \end{array}$$

Experiments are carried out on a preprocessed dataset, and techniques stated above are examined and used. The confusion matrix is used to calculate the performance indicators described above. This matrix describes the model's performance. According to the concept, different algorithms produce different confusion matrixes, as shown in Table 4. Random forest, logistic regression, and naive Bayes classification techniques [43] have been scored for accuracy, as shown in Table 5. Moreover, the random forest has the highest accuracy (99%) among other classifiers and is considered as best suitable choice.

## 5. Conclusion

The number of people dying from heart disease is increasing, making it critical to develop a system that can accurately and efficiently predict heart disease. The study's objective was to find the best effective machine learning method for identifying heart illness. Using data from the UCI machine learning repository, we evaluate the accuracy of logistic regression, random forest, and naive Bayes algorithms for predicting heart disease. As a result of the outcomes of this investigation, the random forest algorithm was determined to have a 99 percent accuracy rate in predicting heart disease which outclasses previously studied models. In the future, we will consider different input features to check the accuracy of existing models.

## Figures and Tables

**Figure 1:** Histogram representation of old peak attribute.

**Figure 2:** Histogram representation of age attribute.

**Figure 3:** Histogram representation of red blood pressure attribute.

**Figure 4:** Confusion matrix representation of random forest and logistic regression.

**Figure 5:** Confusion matrix representation of naïve Bayes.

**Figure 6:** Normalization matrix representation of naïve Bayes.

**Table 1:** Abbreviations and acronyms.

Acronyms	Description

WHO	World health organization
AIRS	Artificial immune recognition system
ML	Machine learning
LR	Logistic regression
RF	Random forest
NB	Naive Bayes
KNN	*k*-Nearest neighbor
CHD	Coronary heart disease risk
NB	Naive Bayes
CANFIS	Coactive neuro-fuzzy inference method
TP	True positive
FN	False negative
TN	True negative
FP	False negative
IoT	Internet of things
ID3	Iterative dichotomized 3
CART	Classification and regression tree

**Table 2:** Machine learning approach to predict heart diseases.

Reference	Method	Accuracy

[1]	Fuzzy-expert system	94%
[28]	Svm, KNN, LG, RF, NB, & LSTM	58%, 76%, 78%, 79%, 82% & 94%
[29]	Hybrid model	85.71%
[30]	KNN with parameter weighting	81.9%
[19]	ANN & BPNN	83%
[20]	LR, RF, NB, GB & SVM	86%, 80%, 84%, 84% & 79%
[21]	NB, SVM & KNN	75%, 45.11% & 50.44%,
[22]	Fuzzy logic	98%
[26]	GUI and WAC	81.51%
[27]	KNN	80%
[31]	CNN-UDRP (KNN, NB)	82%,
[32]	GDB tree algorithm & RF	96.75% & 97.98%
[33]	CSHCP	97%
[34]	CA-SHR	96.02%
[9]	CervDetect	93.6%
[35]	Modified YOLOv5	96.50%
[25]	*K*-means/MAFIA with ID3 & C4.5	89.0% & 81.9%

**Table 3:** Dataset attribute, icon, detail, and range.

Sr. no.	Attribute	Representative icon	Details	Range

1	Age	Age	Patients age, in years	29–71
2	Sex	Sex	0 = female; 1 = male	0,1
3	Chest pain	Cp	4 types of chest pain (1—typical angina; 2—atypical angina; 3—nonanginal pain; 4—asymptomatic)	0,1,2,3
4	Rest blood pressure	Trestbps	Resting systolic blood pressure (in mm Hg on admission to the hospital)	94–200
5	Serum cholesterol	Chol	Serum cholesterol in mg/dl	126–564
6	Fasting blood sugar	Fbs	Fasting blood sugar >120 mg/dl (0—false; 1—true)	0,1
7	Rest electrocardiograph	Restecg	0—normal; 1—having ST-T wave abnormality; 2—left ventricular hypertrophy	0,1,2
8	MaxHeart rate	Thalch	Maximum heart rate achieved	71–202
9	Exercise-induced angina	Exang	Exercise-induced angina (0—no; 1—yes)	0,1
10	ST depression	Oldpeak	ST depression induced by exercise relative to rest	0–6.2
11	Slope	Slope	Slope of the peak exercise ST segment (1—upsloping; 2—flat; 3—down sloping)	1,2,3,
12	No. of vessels	Ca	No. of major vessels (0–3) colored by fluoroscopy	0,1,2,3
13	Thalassemia	Thal	Defect types; 3—normal; 6—fixed defect; 7—reversible defect	0,1,2,3
14	Num (class attribute)	Class	Diagnosis of heart disease status (0—nil risk; 1—low risk; 2—potential risk; 3—high risk; 4—very high risk)	0,1

**Table 4:** TP, FN, FP, and TN rate of RF, LR, and NB machine learning algorithms.

	RF	LR	NB

TP	69	69	69
FN	0	0	0
FP	83	0	0
TN	0	83	83

**Table 5:** Performance of evaluation matrix.

Algorithms	Accuracy	Precision	Recall	*F*1 score

Naïve Bayes	0.97	0.96	0.98	0.99
Logistic regression	0.98	0.99	0.99	0.99
Random forest	0.99	1.00	1.00	1.00

## Data Availability

All data are present in the article.
